The article "Unlocking Early Cancer Detection: Exploring Biomarkers, Circulating DNA, and Innovative Technological Approaches" was retracted in 2025. Reason: concerns about the authorship.

# Unlocking Early Cancer Detection: Exploring Biomarkers, Circulating DNA, and Innovative Technological Approaches

**DOI:** 10.7759/cureus.51090

**Published:** 2023-12-25

**Authors:** B. Krishna Prasanth, Saad Alkhowaiter, Gaurav Sawarkar, B. Divya Dharshini, Ajay R. Baskaran

**Affiliations:** 1 Department of Community Medicine, Sree Balaji Medical College and Hospital, Bharath Institute of Higher Education and Research, Chennai, IND; 2 Department of Gastroenterology, College of Medicine, King Khalid University Hospital, Riyadh, SAU; 3 Rachana Sharir, Mahatma Gandhi Ayurveda College, Hospital and Research Centre, Datta Meghe Institute of Higher Education and Research, Wardha, IND; 4 Department of Biochemistry, Government Medical College, Khammam, Telangana, IND; 5 Department of Psychiatry, National Health Service, Shrewsbury, GBR

**Keywords:** biopsy, early symptoms, early detection, cancer, biomarkers

## Abstract

Research and development improvements in early cancer diagnosis have had a significant positive impact on health. In the treatment and prevention of cancer, early detection is essential. In this context, biomarkers are essential because they offer important information on the state of cells at any particular time. Cells go through unique changes when they shift from a healthy condition to a malignant state, changes that appropriate biomarkers may pick up. Recent advancements have been made to identify and characterize circulating cancer-specific mutations in cell-free circulating DNA derived from tumors and tumor cells. A patient's delay between the time they first detect symptoms and the time they contact a doctor has been noted for many cancer forms. The tumor's location and features significantly impact the presentation of symptoms judged appropriate for early diagnosis. Lack of knowledge of the severity of the symptoms may be one cause for this delay. Our review is largely focused on the ongoing developments of early diagnosis in the study of biomarkers, circulating DNA for diagnosis, the biology of early challenges, early symptoms, liquid biopsies, detectable by imaging, established tumor markers, plasma DNA technologies, gender differences, and artificial intelligence (AI) in diagnosis. This review aims to determine and evaluate Indicators for detecting early cancer, assessing medical conditions, and evaluating potential risks. For Individuals with a heightened likelihood of developing cancer or who have already been diagnosed, early identification is crucial for enhancing prognosis and raising the likelihood of effective treatment.

## Introduction and background

Creating medical diagnostics that can diagnose cancer early or identify its return earlier is a goal that physicians and researchers share with most patients. This shared objective attempts to improve patient prognoses, ultimately raising the possibility of a full recovery. The screening process presents a significant opportunity to detect cancer in its early stages, potentially before the onset of symptoms and ideally before metastasis. This holds for both individuals in good health and those with an elevated risk of the disease. Early cancer identification can lessen the severity of the disease and increase survival rates. Depending on how early the disease's progression is discovered, surgical intervention may be necessary in certain cases as the primary form of treatment. If they could access early detection programs promptly and receive the right care, many cancer patients might be able to reduce suffering and prevent dying too soon. Beyond sociodemographic characteristics like age and socioeconomic standing, factors, including the accessibility of healthcare information regarding cancer indications among the general public and healthcare professionals, particularly those in primary care, impact cancer survival [1]. Access to pertinent diagnostic procedures and efficient medical care is also essential. Early cancer detection depends on spotting symptomatic cases while the disease is still restricted to the organ of origin and not spread to other tissues. Finding substantial cancer or precancerous abnormalities at the earliest possible time, when action might improve survival chances or lessen sickness, is the main objective of early detection. Illnesses that might cause mortality or significant morbidity during the individual's predicted lifespan are called consequential illnesses [2]. Several early detection concepts relate to various facets of cancer treatment, such as the diagnosis of minimum residual disease or the return of the disease. A country must make an impetus effort for early cancer diagnosis as it is essential to all-encompassing national cancer control initiatives. Nonetheless, several essential components exist to consider when encouraging early cancer detection, and this strategy has some drawbacks as well. Early detection results depend on the stage of the disease at the time of a confirmed diagnosis and the start of therapy. When early detection is combined with diagnosing malignancies that have not yet spread far, the benefits can be significant. Furthermore, the time between the development of clinical symptoms and the diagnosis may affect even if early detection is successful. The importance of early detection varies depending on the kind of cancer and its incidence rates. While fast-developing, aggressive tumors often exhibit symptoms earlier than slower-growing, less aggressive tumors, the latter may remain asymptomatic for extended periods. The advantages of early-stage identification for survival may not be as obvious when a significant share of cancers are aggressive [3]. The overall survival statistics are frequently low for certain cancers, including liver cancer, pancreatic cancer, and mesothelioma, regardless of whether the tumor is diagnosed in a localized state. On the other hand, Hodgkin's disease and testicular cancer do not always have inferior survival chances when a disease diagnosis has already reached an advanced stage [4]. Several requirements need to be satisfied for screening to be successful. The targeted cancer must dramatically raise the incidence of disease and mortality. A screening test should be conducted to identify the illness in its early stages and must be validated, safe, and acceptable. It's crucial to comprehend how cancer develops naturally. An identifiable latent or early asymptomatic stage of the malignancy must also be present when no obvious signs or symptoms exist. It is critical that most or all the patients in the preclinical phase move on to the clinical phase without intervention. Consideration should also be given to the problem of *pseudo-cancer* or the possible overdiagnosis of benign illnesses that would never develop into true cancer. For the cases that have been identified, safe and efficient therapies should also be accessible. Additionally, it's important to consider the screening test's cost-effectiveness in proportion to the total amount spent on healthcare. It is critical to be aware of the different screening biases that may influence results when screening people with cancer who have not yet been diagnosed. Early cancer diagnosis has benefited health significantly because of research and technological advances. This is demonstrated by the fact that tumors with established screening regimens, such as cervical, breast, and colorectal cancers (CRCs), have fewer cases of advanced diagnosis than cancers without such protocols [5]. Lead-time bias is a risk factor for screening because it can affect the timing of a cancer diagnosis without changing the final result. While screening, there is also a risk of overdiagnosis when early invasive or potentially precancerous lesions and malignancies are discovered that did not necessitate treatment over the patient's lifetime. Increasing early cancer diagnosis has the potential to raise survival rates dramatically. Although recent improvements in early detection have helped save lives, continued research and the innovation of fresh methods for early cancer diagnosis are still essential. In addition to utilizing technical breakthroughs for breast cancer testing in females with a hereditary risk for the disease or who may have one, the American Cancer Society (ACS) is currently investigating testing methods for CRC using stool samples [6]. These updates act as guidelines for averting and promptly identifying skin cancer. Early detection aims to spot significant cancer or precancerous alterations as early as feasible to improve survival or lower morbidity. In this context, *consequential diseases* refer to illnesses expected to cause death or serious health problems during a person's estimated lifespan. Several facets of cancer care, such as the discovery of minimal residual illness or a return of the disease, are also impacted by the concepts of early detection. Research and development improvements in early cancer diagnosis have had a significant positive impact on health. Notably, compared to cancers lacking screening procedures, cervical, breast, and CRCs have established screening approaches that have decreased the prevalence of later-stage diagnosis. Modern imaging techniques have limitations since they can only detect cancers with more than 10 cells and may not detect smaller or earlier-stage tumors. CT scans with minimal radiation exposure for detecting lung cancer, in its initial stages of identification in high-risk populations, and tissue morphology imaging are used in breast cancer screening using X-ray mammography [7]. Molecular imaging tools, such as magnetic resonance imaging (MRI) modules, enable early diagnosis and staging. Time-of-flight positron emission tomography (PET) scans, for instance, represent well-known versions of these technologies that can provide enhanced sensitivity, specificity, or positive predictive value. Radiologists are greatly aided by computer-assisted diagnostic tools when evaluating medical pictures. Furthermore, computer-driven feature extraction can take advantage of texture and form variations invisible to the unaided sight. Another new technique is photoacoustic imaging, which involves shining pulsed laser light at a particular wavelength on the region of tumors to produce sound waves that may be detected by piezoelectric or microphone sensors [8].

## Review

Biomarkers

Biomarkers have various uses, including identifying illness early in individuals who might not show symptoms, diagnosing diseases in tissue samples, and monitoring patient response to treatment. Diagnostic markers can non-invasively identify early-stage cancers, enabling the start of therapy when the condition is still treatable. Applying classification algorithms to find changes in marker levels related to illness state is the first stage in the development of biomarkers. It is important to note that identifying these markers frequently depends on data-driven methods instead of being founded on predetermined biological ideas. More potential markers may be found if biological factors are better included in the marker-finding process [9]. In addition to the conventional diagnostic techniques, screening programs within the investigation can be utilized on the target population to study novel disease indicators. To ensure proper laboratory procedures in marker research, strict standard operating procedures must be followed, sample analyses must be performed without awareness of the presence of any diseases, and batch effects must be minimized [10]. When seen alone, biomarkers can occasionally look binary or categorical, but their usefulness gives prognostic and useful information that guides therapeutic decision-making. Early cancer indicators include biochemical abnormalities and visible structural changes in the tissue. Frequent sampling from healthy people and those at risk is necessary, and least intrusive sampling techniques are recommended wherever possible because proteomics reflects both the underlying cell's DNA code and the effects of the immediate atmosphere [11]. Transcription, post-transcriptional alterations, and translational events are a few examples of the mechanisms that can control the production and function of proteins. As a healthy cell changes into a neoplastic cell, several obvious changes occur at the protein level. Changes in protein expression, differences in protein modifications, variations in certain protein functions, and atypical changes in protein localization are all included in these alterations. Collectively, these changes may affect the well-being of cell functions overall. The recognition and understanding of these alterations are the primary goals of cancer proteomics. Cancer proteomics research aims to identify biomarkers that help early cancer identification and select the most effective therapy approaches.

High levels of cancer biomarkers may indicate cancer, but other conditions may also cause them. It is important to discuss the results of a cancer biomarker test with a doctor to determine what they mean for the individual patient (Table 1).

**Table 1:** Commonly employed tumor markers for screening and monitoring. Source:  [12]. CA 125, cancer antigen 125

Biomarker	Cancer type	Associated biomarkers	Clinical significance
Alpha-fetoprotein	Germ cell tumors	Hepatocellular carcinoma	High levels may indicate cancer.
Beta-human chorionic gonadotropin (beta-hCG)	Malignant tumor of trophoblastic tissue	Cancer affecting the testicles	High levels may indicate cancer.
Beta-2 microglobulin (β2-M)	Plasma cell myeloma	Persistent lymphocytic leukemia	Lymphomas
CA 125	Ovarian	CA 125 is often used as a stand-alone biomarker for ovarian cancer screening.	High levels may indicate cancer.
CA 15.3 and CA 27.29	Breast	CA 15.3 and CA 27.29 are associated with breast cancer.	High levels may indicate cancer.
CA 19.9	Pancreas	Gallbladder and bile duct	May indicate pancreatic, gallbladder, or bile duct cancers.
CD20	Non-Hodgkin lymphoma	β2-M and lactic dehydrogenase	High levels may indicate cancer.
Calcitonin	Medullary thyroid	RET proto-oncogene mutations	High levels may indicate cancer.
Carcinoembryonic antigen	Ovarian, cervix, and breast	Associated with ovarian, cervix, and breast cancers	May indicate cancers in the ovaries, cervix, or breast.
Lactate dehydrogenase	Germ cell tumors	Associated with cellular damage and not exclusive to germ cell tumors	High levels may indicate cancer.
Prostate-specific antigen	Prostate	Prostate cancer	High levels may indicate cancer.

Circulating DNA (ctDNA)

Due to recent significant advancements in the identification and characterization of circulating tumor cells (CTCs) and cancer-specific mutant cell-free ctDNA, it is now feasible to use these cancer screening tests. It is crucial to remember that CTCs and ctDNA have yet to establish standards in common clinical practice. The capacity to separate tumor cells, permitting both morphological identification and molecular analysis, is a major benefit of using CTCs in cancer care. CTCs and ctDNA have demonstrated predictive importance in cases of advanced illness across various tumor types [13]. Additionally, early markers of treatment response might be the first shifts in marker levels throughout therapy. The accuracy of any cancer screening test is essential since false-positive findings can cause patient concern and call for more testing, which is expensive and could have negative health effects [14]. The release of mutant DNA seems to occur exclusively within the bloodstream when a tumor is invasive and usually does so through apoptosis or necrosis, ctDNA, in particular, should have great specificity. More than 80% of advanced tumors, including those where CTCs cannot be detected, and ctDNA also offers increased sensitivity.

Biology of early challenge

Understanding the basic mechanisms in the early stages of cancer reveals a progressive change from a healthy condition to a dysregulated one and finally to a malignant state. Developing a thorough knowledge of this biology will enable us to predict the future path of these changes. Minor dysregulations in molecular and cellular features mark the initiation of cancer. As the process develops, the cell's genome or epigenome significantly changes, leading to malignant transformation. A distinctive collection of aberrant characteristics of cancer results from this transition [15]. The cancer might then progress to potentially end stages of metastasis and invasion into nearby tissues. The dynamics of the illness are further complicated by the fact that cancer cells continue to develop and diversify during this process. Understanding this timeline might help determine the best window for discovery and intervention because the transition rate between different stages depends on the specific form of cancer. A phylogenetic tree could be used to pinpoint the genesis of a malignancy in a specific cell [16]. This single cell forms under particular circumstances and is regulated by the tissue microenvironment and the immune system. It's crucial to remember that each organ system offers a unique environment, and some mutations may result in a potentially fatal tumor in one organ setting but not in the other. A tumor-permissive environment can be created by variations in non-cancerous cells brought on by aging, such as biophysical changes in the extracellular matrix, changes in secreted substances, and adjustments to the immune system [17]. The cellular microenvironment substantially impacts the transition from a healthy cellular state to a malignant one. The extracellular matrix, vascular cells, host immune cells, supporting mesenchymal cells, and secreted proteins are a few components that make up this milieu. It may live in various pH ranges and hypoxic (low oxygen) circumstances [18]. A prospective tumor cell's unique microenvironment may be crucial to the development of the tumor, ultimately dictating whether the cell stays isolated or aggressively spreads. Additionally, early tumor growth might lead to changes in the microenvironment that could cause measurable modifications and act as biomarkers for early diagnosis (Figure 1).

**Figure 1:** The timely identification of cancer. Image credit: B. Divya Dharshini.

Early symptoms

Although there is a well-established staging system for dividing cancer into early and advanced stages, it is critical to remember that the terms *early* and *advanced* when referring to cancer signs and symptoms are not consistently and precisely used by healthcare professionals and can vary between countries. The tumor's location and features significantly impact the presentation of symptoms judged appropriate for early diagnosis. Specific symptoms only might sometimes show up once the disease has progressed further. There are currently few definitions of early signs of cancer that are exact, generally relevant, and included in medical textbooks or national recommendations. Following the presentation of initial symptoms frequently, primary care providers come across patients experiencing hematuria, hemoptysis, dysphagia, and rectal bleeding; there is a noticeably increased risk that certain cancer types (such as urinary tract, respiratory tract, esophagus, and colorectal) would be discovered [19]. Table 1 covers malignancies based on the most recent medical data, reference materials, medical literature, etc. Early diagnosis and the manifestation of observable medical signs, commonly linked with an earlier presentation in cancer patients, are crucial. Cancers that develop indications in a later stage of the illness and, as a result, have worse relative survival rates, on the other hand, are less accessible to early detection. Table 1 lists the malignancies for which early detection is crucial and the clinical signs frequently present at the earlier presentation of cancer patients. Lung malignancies stand out because they frequently exhibit inexplicable or recurrent symptoms such as chest discomfort, dyspnea, hoarseness, clubbing of the fingers, coughing up blood, and trouble breathing. Liver malignancies often have dismal survival rates when there are no obvious symptoms [20]. It frequently means that the illness has advanced when symptoms like hypoglycemia, intraperitoneal hemorrhage, high serum alpha-fetoprotein levels, ascites (abdominal fluid buildup), or hepatomegaly (enlarged liver) appear. Similar patterns have been seen in upper gastrointestinal tract tumors, including stomach cancer. Unexpected weight loss, upper abdominal discomfort, the appearance of indications in a later stage of the condition, and trouble swallowing are among the symptoms most commonly associated with these tumors [21].

Liquid biopsies

Examining CTCs DNA from tumors in circulation or extracellular vesicles derived from tumors released into the circulation from tumors and their metastatic locations constitutes the basis of *liquid biopsies*. Comprehensive reviews on CTCs, ctDNA, and extracellular vesicles have already been published [22]. Liquid biopsies, which analyze physiological fluids, can identify several cancer-indicative chemicals. These compounds can result from the tumor's existence or the tumor itself. For instance, cell-free DNA (cfDNA), which consists of nucleic acid fragments, enters the circulation after cellular apoptosis or necrosis. A fraction of this ctDNA, which is present in cancer patients, comes from the tumor. For individualized mutation profiling and the monitoring of patients with advanced malignancies, ctDNA analysis shows the existence of tumor cells [23]. In liquid biopsy technologies, there are distinct considerations when applied to precancers and the early stages of neoplastic development compared to their application in advanced cancers. These disparities are crucial in understanding their utility and potential clinical significance. In precancers and early stages, lesions are typically small, often measuring less than 1 cm^3^, while in advanced cancers, lesions tend to be significantly larger, equal to or greater than 1 cm^3^ in size [24]. The substantial size difference can impact detection and diagnostic approaches.

Clinical signs

Clinical signs are usually absent in precancers and early stages, making diagnosis challenging without specialized tests. In contrast, advanced cancers often manifest apparent clinical signs and symptoms, aiding their recognition. Conventional imaging techniques often do not detect these lesions in precancers and early stages. In contrast, advanced cancers are frequently identifiable through imaging due to their size and localization. The biology of precancerous and early-stage lesions varies widely, ranging from favorable to unfavorable, with some precancerous lesions potentially evolving toward malignancy [25]. In contrast, advanced cancers generally exhibit unfavorable (sub) clones, which are more challenging to treat.

Established tumor markers

Identifying well-known tumor biomarkers, such as prostate-specific antigen (PSA), carcinoembryonic antigen (CEA), and cancer antigen 125 (CA 125) in precancers and early stages is uncertain, and even if present, they lack high specificity and sensitivity [26]. In advanced cancers, these markers are frequently available but may still have limitations in terms of specificity and sensitivity. They are often used for disease monitoring rather than definitive diagnosis.

Knowledge of target genes

In liquid biopsy assays, the genes to be targeted are often unknown for precancers and early stages. In contrast, for advanced cancers, these genes are typically recognized or ascertainable through the tumor tissue currently accessible, aiding in assay design and interpretation.

Driver genes

The identity of established driver genes is frequently unknown in precancers and early stages, while in advanced cancers, driver genes are usually known. This knowledge is critical for targeted therapies. Recognizing signs of positive selection and separating them from passenger mutations are important goals in identifying these driver genes. A cancer driver gene is one whose mutations promote net cell proliferation in vivo under particular microenvironmental circumstances. Although the number of driver genes is fewer than 19,000, the entire number is unknown. The criteria used to determine whether a gene is functional have been improved through ongoing study. This improvement has led to various *significantly mutated gene* techniques, which combine more complex metrics of mutational base contexts and account for factors like replication time and gene expression. Instead of establishing if the reported mutation rate of a gene in malignancies is higher than anticipated by chance, ratio metric approaches, which examine the composition of mutations normalized by the total mutations in a gene, are an alternate way of discovering cancer drivers [27].

Plasma DNA technologies

Liquid biopsy assays in precancers and early stages often involve focused high-sensitivity approaches, while in advanced cancers, a broader range of targeted and untargeted techniques are applicable. Fine-needle aspiration, mammograms, ultrasound, and tumor biopsies are essential for a definitive diagnosis. Therefore, having a marker that can evaluate the risk of breast cancer using a straightforward, noninvasive manner would be advantageous for people at risk. DNA damage is a common occurrence and is a constant struggle throughout life. Under unfavorable circumstances like cancer and inflammation, DNA damage occurs more often. DNA repair enzymes can reverse most DNA damage. However, these mechanisms are not always effective. As a result, nuclear-free DNA has been made available in the plasma of cancer patients as a tool for identifying and monitoring cancer [28]. Additionally, plasma DNA offers diagnostic benefits in screening due to its high sensitivity and specificity when used with the fluorometric technique. The amount of plasma DNA in patients with breast cancer may be measured using a commercial kit extraction and a portable fluorometer [29]. Comparing blood sampling to operations like bone marrow aspiration, the former is more practical and less uncomfortable. Therefore, large-scale research must be conducted to clarify early breast cancer identification and recurrent surveillance, including breast cancer patients and healthy controls.

Proximal sampling

Proximal sampling is feasible in precancers and early stages only if the endangered tissue is known, which limits its applicability. In selected advanced tumor entities, proximal sampling is possible but frequently unnecessary. Proximal sampling obtains body fluids other than blood, such as urine, saliva, sputum, cerebrospinal fluid, pleural effusions, and feces. These fluids serve as additional or substitute sources of tumor DNA for liquid biopsies. Their analysis is frequently restricted to identifying local tumors, except urine, where the proximity or direct interaction of the diseased organ with the body fluid may raise the yield of tumor DNA in contrast to systemic sources [30]. Due to the scarcity of ctDNA in these patients' blood, cerebrospinal fluid (CSF) is becoming significant as a source of ctDNA for cancers limited to the central nervous system (CNS) [31]. Lung cancer diagnosis and patient categorization using sputum-derived DNA is becoming increasingly common. A recent study has confirmed the utility of feces-derived DNA as a CRC diagnostic tool, and pancreatic cancer detection has also shown promising results [32]. Urinary DNA has significant importance as a liquid biopsy for various malignancies, including the prostate, intestine, and pelvis, as well as non-urogenital malignant tumors such as non-small cell lung cancer (NSCLC), colon cancer, and stomach cancer [33].

Somatic mutation variant allele frequency (VAF)

VAF is the ratio of mutant molecules to all the wild-type molecules at a certain genomic region. Utilizing cell-free circulating DNA offers a minimally invasive way to evaluate patients with metastatic cancer's mutational status fully. cfDNA somatic mutations can arise from metastases and the main tumor, providing a more thorough understanding of tumor heterogeneity. Additionally, somatic mutations in cfDNA may be caused by clonal hematopoiesis [34]. Precision oncology for cfDNA testing provides a rapid and less invasive method for genomic profiling in advanced/metastatic illnesses. This assists in choosing a course of therapy, acts as an early indicator of response, and keeps track of developed resistance mechanisms. A larger maximal VAF is inversely connected with prognosis and overall survival and partially acts as a proxy for tumor load. VAF, the number of changes, and overall survival to determine if a patient's prognosis is acceptable for clinical trial enrollment. In blood samples, somatic mutations' expected VAF is extremely low in precancers and early stages [35].

Tumor heterogeneity

Tumor heterogeneity is relatively low in precancers and early stages but significantly higher in advanced cancers [36]. Subclones with innate or acquired resistance may be preferred when heterogeneous cancers are exposed to selection forces like drug therapy. These clones of cells can become dominant inside a tumor mass due to this selection. In *liquid biopsies in early screening* or *tumor sampling*, CTCs or cell-free tumor DNA from cancer patients' peripheral blood are examined. For the analysis of primary and metastatic cancers, this kind of sampling offers a reasonably straightforward and noninvasive method [37]. Intra-patient CTC heterogeneity, however, may even represent an obstacle when the objective is the development of a biomarker. Consequently, the search for CTC-based biomarkers needs to be addressed to investigate commonalities in groups with different outcomes rather than differences in single CTCs in CTC pools isolated from different patients. While DNA's fragmented and diluted form makes ctDNA analysis difficult, it is a perfect *liquid biopsy* technique inside wild-type cfDNA. This method enables the minimally invasive surveillance of tumor existence and size, observation of changes in tumor dynamics in response to therapy, identification of actionable genetic mutations, detection of minimum residual disease, and tumor heterogeneity (Figure 2).

**Figure 2:** Heterogeneity within tumors and the evolutionary process at the clonal level. Image credit: B. Divya Dharshini.

Established clinical guidelines

No clinical guidelines exist for liquid biopsy use in precancers and early stages. In contrast, emerging guidelines for patients with NSCLC and blood-based companion diagnostic testing for epidermal growth factor receptor (EGFR) mutations are currently used, with potential uses for advanced malignancies. Advanced liquid biopsy techniques are used differently when detecting precancerous diseases and early neoplastic stages than when treating more advanced tumors. Lesion size, clinical manifestations, detectability, biological traits, target genes, driver genes, DNA release, assay technologies, sampling techniques, customization, VAF, tumor heterogeneity, confounding mutations, and clones; somatic copy number alterations (SCNAs); and adherence to clinical recommendations are a few examples of the factors that are critical in making these distinctions. These factors influence these approaches' therapeutic relevance and efficacy. The ACS's decision to support monthly breast self-examination (BSE) beginning at age 20 is a major development. The amended advice instead strongly emphasizes the value of educating women about the BSE's possible benefits, limitations, and dangers. Women are now urged to decide whether to conduct BSE regularly or irregularly [38]. The ACS advises commencing cervical cancer screening at a maximum age of 21 and approximately three years following the beginning of vaginal sex. It is recommended to undergo routine screening every year until 30 or every two years if utilizing liquid-based cytology. The ACS amended its recommendations in 2002, emphasizing early detection and follow-up for colorectal and adenomatous polyps. Immunochemical assays are now part of the updated guidelines for detecting hidden blood in fecal samples. The ACS suggests that those with an average risk start CRC screening at age 50 [39]. In addition, the U.S. Preventive Services Task Force (USPSTF) advises doctors to check patients 50 and older for CRC. According to the USPSTF's evaluation, several screening techniques effectively lower CRC mortality rates, including colonoscopy, double-contrast barium enema, flexible sigmoidoscopy, and fecal occult blood testing (FOBT) [40]. Due to numerous circumstances, the ACS has found inadequate evidence to support the recommendation of endometrial cancer screening in women at average risk or those at greater risk. These include a history of unopposed estrogen medication, tamoxifen therapy, late menopause, null parity, infertility or inability to ovulate, obesity, diabetes, or high blood pressure. A high probability of carrying a mutation (i.e., a confirmed mutation within the family) or the lack of genetic testing results in families with a potential autosomal dominant colon cancer predisposition may be associated with a significantly elevated risk of developing endometrial cancer in some women. The ACS recommends that males aged 50 or older with a minimum 10-year life expectancy receive a yearly digital rectal exam and PSA test. Men should be informed of the benefits and restrictions of early diagnosis and treatment for prostate cancer before agreeing on testing. A doctor must help people make educated decisions. Men with a greater risk should start testing at age 45, including those of sub-Saharan African origin and those with a first-degree relative diagnosed before age 65. For people with a higher risk due to having several relatives who were identified at 65, testing before age 40 may be considered [41].

Gender differences

Compared to women, men have greater incidence and fatality rates from cancer. While their underuse of primary preventive methods is the main cause of this imbalance, gender disparities in early detection procedures may also play a role. The discrepancies in death rates might be attributed to gender-specific variations in screening process adoption or the prompt identification of symptoms. Self-examination is commonly encouraged for visible or palpable tumors, such as cutaneous, testicular, and breast malignancies. For instance, skin self-examination may cut melanoma-related mortality by as much as 63% [42]. Early research indicates that men are less inclined than women to do self-reflection. Women are better at finding melanoma on themselves, and wives are noticeably better at finding melanoma on their husbands than the opposite is true [43]. Encouragement of people, particularly men, to actively look for signs seems more difficult. Compared to men's understanding of testicular self-examination, women frequently demonstrate increased awareness of BSE, and more women report doing so. This lower rate of self-examination among males may be a sign of a larger discrepancy in perceived vulnerability and health awareness. In addition, gender biases in healthcare personnel' attitudes and behaviors could have an impact. A patient's delay between the time they first detect symptoms and when they contact a doctor has been noted for several cancer forms. Lack of knowledge of the severity of the symptoms may be one of the causes of this delay. There are not many reports of lengthier delays in males, notwithstanding the paucity of evidence on gender differences in this area. Contrarily, it has been found in several CRC research that males are more reluctant to delay seeing a doctor after developing symptoms [44]. Men typically have a more limited understanding of cancer symptoms than women. According to trends seen in primary prevention regarding the utilization of healthcare services and adherence to healthcare practices, the gender disparity in engagement with screening programs is most pronounced prominent among younger age groups. Individuals' judgments of the significance of taking preventive measures, their assessments of disease risk, and their evaluations of the advantages and disadvantages of cancer testing are only a few of the variables that affect cancer detection and prevention practices. Generally, men tend to place less importance on health protection strategies and report lower frequencies of such practices [45]. ​​​​​​

Instructions for spotting early signs

FOBT is not as sensitive as fecal immunochemical testing (FIT) for detecting CRC. Flexible sigmoidoscopy is not as sensitive as colonoscopy for detecting CRC (Table 2).

**Table 2:** Suggestions by the American Cancer Society for identifying cancer at an early stage in asymptomatic individuals with a typical risk profile. Source: [46]. FOBT, fecal occult blood testing; FIT, fecal immunochemical test; DRE, digital rectal examination

Cancer location	Sex	Age (years)	Diagnostic test	Occurrence rate
Breast	Women	20	Breast self-examination	Commencing during their initial twenties
Breast	Women	20	Clinical breast examination	Once every three years for women in their twenties and thirties and on an annual basis for women aged 40 years or above
Breast	Women	40	Mammography	Annually
Intestinal and rectal	Men/Women	50	Testing for hidden blood in the stool, either through FOBT or FIT	Annually
Colorectal	Men/Women	50	Flexible sigmoidoscopy, or	Every five years
Gastrointestinal and rectal	Men/Women	50	Testing for hidden blood in stool (FOBT) and flexible sigmoidoscopy	Each year and at intervals of five years, respectively
Colorectal	Men/Women	50	Double-contrast barium enema	Every five years
Colorectal	Men/Women	50	Colonoscopy	Every 10 years
Prostate	Men	50	Examination of the rectum through digital means (DRE) and the measurement of prostate-specific antigen (PSA) levels	Annually
Cervix	Women	18	Pap test	Every year (conventional) or every two years (liquid-based)
Cervix	Women	30	Pap smear or human papillomavirus DNA test in conjunction with cervical cytology	Either every two to three years with a Pap test or every three years with a combination of a human papillomavirus DNA test and cervical cytology
Endometrial	Women	Menopause	Medical examination for cancer-related concerns	During a routine health checkup

Guidance for women with an average risk of breast cancer

Women highlight a procedure that starts when a woman reaches age 20 and entails a mix of clinical breast examinations, education about breast symptoms, and routine mammography commencing at 40 years. Women are advised to undergo clinical breast exams, beginning at age 20, continuing until age 39, and then annually thereafter, with exams performed every three years. This examination allows medical personnel to evaluate the patient's family history of breast cancer, making it an essential part of regular health exams. It opens up the topic of early detection for conversation, emphasizes the value of commencing routine mammograms at age 40, and responds to any queries or worries that women may have about their particular risk and new early detection methods or related topics. Women should know BSE's potential advantages, restrictions, and negative effects. The ACS advises average-risk women to start yearly, initiating mammography screening at 40 [47]. Women should also be made aware of the limits of mammography, particularly the fact that not all breast cancers can be discovered by the procedure and that some of those can still have a bad prognosis. The ACS's recommendations for cervical cancer screening are consistent with the general understanding concerning the epidemiology of cervical intraepithelial neoplasia, particularly the contributing role of the human papillomavirus [48]. These guidelines suggest several monitoring strategies depending on a woman's age, screening history, and preferences for screening and diagnostic technology. Before becoming 21, the ACS advises beginning a cervical cancer screening program, but no later than three years following the first vaginal encounter. Women with moderate risk should undergo annual cervical cytology smears between the ages of 30 and 70 or opt for biennial liquid-based cytology screenings. Women over the age of 70 who still have an intact cervix may decide to stop getting screened for cervical cancer, if there is proof of three consecutive technically adequate and normal test results for those in this risk category, provided they have not had any abnormal or positive test results in the 10 years before turning 70. For people who have a higher-than-average risk of getting colon cancer, the ACS advises increased surveillance. This includes those who have adenomatous polyps, a history of CRC that was successfully removed surgically, a family history of the disease, and colon adenomas that were discovered in a first-degree relative under the age of 60, as well as people who have a long history of inflammatory bowel disease, are among those who fall into this higher-risk category [49]. At the start of menopause, women with ordinary to higher risk profiles must be made aware of the warning signs and symptoms of endometrium cancer, especially sudden bleeding and spotting. It is crucial to emphasize the importance of treating these symptoms seriously and swiftly alerting medical professionals. The most common way to collect endometrial tissue is still endometrial biopsy, and the standard method for determining the health of the endometrium is still endometrial histology analysis, despite continuous research into different ways [50]. The ACS suggests commencing the PSA and digital rectal examination (DRE) yearly at age 50 for males, with a life expectancy of at least 10 years. This should be followed by discussing the potential advantages, restrictions, and disadvantages of testing [51].

Breast cancer

BSE can be regarded as a part of breast cancer screening. Still, when they approach the age of 40, it's vital also to have a medical professional doing clinical breast exams expert every three years. Women should be urged to tell their doctors when they notice any changes in their breasts. Early breast cancer detection is greatly aided by mammography. A 19% decrease in breast cancer mortality is linked to routine mammography screening, with a roughly 15% decrease for women in their forties and a 32% decrease for those in their sixties [52]. Based on a person's potential for breast cancer development and knowledge of the possibility of false-positive results, it is important to carefully examine the age at which mammography should start and how frequently it should be performed. Organizations advise mammography tests for women between 50 and 70 years at least every two years; however, some urge yearly screenings beginning at age 40 [53]. It is critical to recognize that mammography has the risk of false-positive findings and can result in overdiagnosis. To make an informed choice, one should consider family history, personal preferences, individual risk, and professional suggestions. The variability among radiologists has been reduced, the detection rates for breast cancer have increased, and several artificial intelligence (AI) algorithms have been created specifically for screening mammography. Google's AI system analyzes computed tomography (CT) images to determine the likelihood of lung cancer. However, solutions depending on MRI, CT scans, or mammography may be limited in environments with low resources. Consequently, there is a need for mobile AI-based screening solutions that rely on something other than heavy, expensive infrastructure. As a result, preventive screening would become more affordable, practical, and accessible (Figure 3) [54].

 

**Figure 3:** A diagram of the causes of radiation exposure in breast cancer screening. Image credit: B. Divya Dharshini.

Colorectal cancer

Numerous surveillance studies conducted over the last four decades have provided evidence to support the concept that CRC’s early identification improves clinical outcomes. The National Polyp Study from 1978 showed that eliminating adenomatous polyps greatly lowers the incidence of CRC [55]. Adenomatous polyps are precursors of CRC. More recent population-based studies have also shown a significant decrease in CRC risk and death linked to routine colonoscopy examinations. Case-control, cross-sectional, and cohort approaches were employed in this research. Notably, compared to the proximal colon, the protective benefits of colonoscopy screening are more prominent in the distal colon. The National Comprehensive Network for Cancer advises CRC screening for people with no personal or family adenomas, CRC sessile serrated polyps (SSPs), or inflammatory bowel disease in the past should begin at age 50 [56]. Rescreening with any screening method is advised after 10 years. Colonoscopy examination for hyperplastic, polyps, or non-SSP lesions less than 1 cm is critical [57]. If the sigmoidoscopy results are negative, people should be reevaluated five years later using any screening technique. However, if adenomas or SSP lesions are seen, planning a follow-up colonoscopy every two to six months or three or five years, depending on the precise findings, is crucial. The frequency of the subsequent colonoscopy varies on parameters, including the resection's quantity, size, and completeness. A comprehensive screening program targeted at early diagnosis and polyp removal will most benefit patients at a higher risk of developing hereditary CRC [58]. Individuals at high risk should think about getting a colonoscopy every one to two years, starting at age 25 to 30 or two to five years before they are diagnosed with colon cancer if it develops before age 30. Starting at the age of 10 to 15, it is advised that people with familial adenomatous polyposis (FAP) who have an adenomatous polyposis coli (APC) mutation have flexible sigmoidoscopy or colonoscopy performed every 12 months. As they age, the idea of a preventative colectomy is something to consider [59]. Colonoscopies for those with juvenile polyposis syndrome (SMAD4 mutations) should start around age 15 and be done yearly if polyps are found or every two to three years if none exist. Upper endoscopy is advised to use a similar strategy. Starting at the age of 10 to 15, it is advised to have a flexible sigmoidoscopy or colonoscopy performed every 12 months for people with FAP caused by an APC mutation [60]. When they are adults, preventive colectomy should be taken into account. Colonoscopy should start at age 15 and be performed annually if polyps are detected or every two to three years if none are found for those with juvenile polyposis syndrome (SMAD4 mutations). For upper endoscopy, a similar strategy is recommended [61].

Technologies

The problem of creating technology with great sensitivity for identifying even the smallest cancers while reducing false positives is a crucial one. Most imaging methods now being used in clinical settings or being developed cannot identify such tiny cancers [62]. However, in vivo imaging technology is always improving, as demonstrated by the 10.5T MRI, which continually pushes the limits of detection. Another potential strategy is activity-based diagnostics, which uses enzyme activity to create exogenous biomarkers indicating cancer. For instance, scientists have developed nanoparticles that preferentially cleave when protease activity is dysregulated in cancer cells, producing urine reporters. Innovative methods have arisen in synthetic biology, such as immune cell diagnostics and customized probiotics intended for tumor detection via amplified, activity-based readouts. Significant advancements in material engineering and microfabrication have also contributed to creating devices that may mimic physiological microenvironments [63]. These tools make it possible to study the biology of tumors and separate extracellular vesicles and CTCs from patient samples.

AI in diagnosis

Histopathology is a crucial stage in early detection for confirming the diagnosis and offering prognostic information after the first identification using biomarkers and/or imaging. The combination of digital pathology with AI can improve the accuracy of diagnostic evaluations, identify early signs of cancer, and provide useful information for research [64]. However, digital pathology also needs help, such as dealing with artifacts, controlling sample variances, needing more binary variables when a diagnosis can call for a risk assessment, and blending samples from various populations and locales. Many biological markers were created for cancer for several objectives, including staging, prognosis, and therapy selection. It could be more prudent that few recognized diagnostic indicators perform well enough to be used in asymptomatic groups. Identifying early-stage cancer using biomarkers in physiological fluids at low quantities is difficult while retaining a high degree of specificity equivalent to imaging methods [65]. It is frequently required to collect pre-diagnostic samples from people who acquire the disorder with relevant markers. Traditional case-control studies find it difficult to get such samples, but alternative prospective research methodologies might be used. It is critical to incorporate biomarker research into these resource-intensive longitudinal studies, using them as platforms by advice from groups like the Early Detection Research Network (EDRN) and expert perspectives. Increased cooperation between epidemiologists and laboratory teams is required to improve the quality of screening initiatives, nationwide cohort studies, and randomized controlled trials targeted at finding and verifying markers. Detecting asymptomatic illnesses with diagnostic markers requires extremely high test specificity to save clinically healthy people from intrusive diagnostic procedures. Achieving a level of specificity comparable to imaging techniques is a formidable task for biomarkers, such as the 98% specificity of mammography [66]. Developing decision algorithms to evaluate the evidence for positivity is also necessary since panels of concurrent testing may produce an accumulation of false-positive findings. After a positive result, implementing a timely second screening or a progressive approach to further testing might help lower false positives to a manageable level. Point-of-care tests may be used for the first round of widespread screening, and for individuals who test positive, more complex assays may be used. As shown by the cautionary example of PSA, straightforward diagnostics must only enter clinical practice after they get enough validation. However, inpatient cohorts being watched for illness recurrence may be exceptions to the rigorous standard for high specificity in diagnostic markers. Diagnostic marker screening only applies to surrogate tissues, such as blood feces, because invasive tissue urine collection techniques are impractical for the target organs of asymptomatic persons [67]. Consequently, imaging techniques unique to the target organ have become essential tools.

## Conclusions

In summary, with growing biological understanding and technical improvements, early cancer detection research is at a critical juncture. It is getting closer to its goal of promoting early curative therapies and higher cancer survival rates. Despite these obstacles, early cancer diagnosis is becoming acknowledged as a critical area for public health advancement. The assessment suggests a framework to hasten the development of this area. Integrating biology, clinical expertise, technology, data analysis, risk assessment, and health system research requires interdisciplinary collaboration. To have a meaningful impact on survival rates, early detection must be seamlessly integrated into healthcare systems, leading to evidence-based interventions that can prevent cancer progression or lead to a cure. Other crucial objectives include ensuring equity, accessibility, and minimization of damage. The review goes through the value and difficulties of early cancer detection. While early detection of cancer is essential for improved outcomes, there is a potential for overdiagnosis and overtreatment, as well as the fact that early detection does not necessarily mean a higher probability of a cure.
